RETRACTED

# Activating IL-6/STAT3 Enhances Protein Stability of Proteasome 20S *α*+*β* in Colorectal Cancer by miR-1254

**DOI:** 10.1155/2022/4250013

**Published:** 2022-05-14

**Authors:** Weiguo Ren, Xuexiu Zhang, Qiang Li, Chibin Pu, Decai Zhang

**Affiliations:** ^1^Department of Gastroenterology, The First Affiliated Hospital of Zhengzhou University, Zhengzhou, Henan 450003, China; ^2^Oncology Department, Shenzhen Hospital, Southern Medical University, Shenzhen, Guangdong 518101, China; ^3^Department of Gastroenterology, Zhongda Hospital, Southeast University, Nanjing, Jiangsu 210009, China; ^4^Department of Gastroenterology, The Third Xiangya Hospital of Central South University, Changsha, Hunan 410000, China

## Abstract

A widely recognized feature of colorectal cancer (CRC) is an increase in cytokine levels, which result in an inflammatory environment in the tumor. Interleukin-6 (IL-6) is a robust protumor cytokine. Several studies suggest that IL-6 plays a role in the development of tumors. Most intracellular protein breakdown occurs in eukaryotes via the ubiquitin-proteasome pathway; this mechanism may also be involved in cancer pathogenesis. The tumor tissues and paracancerous tissues were collected from 90 patients with colorectal cancer. The expressions of pSTAT3, proteasome 20S *α*+*β*, miR-1254, and PSMD1 in tissues were detected by immunohistochemistry, ELISA, and qRT-PCR, and the effects of pSTAT3 and proteasome 20s *α*+*β* expressions on the survival of patients were studied. HCT116 and HCT116-R cells were cultured and added IL-6, AG490, STAT3 plasmid, or overexpression/knockdown of miR-1254 in cells. Immunofluorescence, western blot, qRT-PCR, double luciferase gene reporter assay, and flow cytometry were used to detect the expression of pSTAT3, STAT3, proteasome 20s *α*+*β*, miR-1254, and PSMD1 and cell cycle. The nude mouse xenograft model was constructed and divided into 3 groups: PBS group, IL-6 treatment group, and IL-6+miR-1254 mimic group. After 28 days, the tumor tissues were collected, and the expressions of miR-1254, pSTST3, proteasome 20s *α*+*β*, and PSMD1 in the tissues were detected by qRT-PCR and immunohistochemistry, respectively. Our study discovered that the level of proteasome 20S *α*+*β* had a strong connection with pSTAT3 in CRC patients. They were also linked to the development and clinical outcome of CRC. In addition, we found that IL-6 dramatically increased the expression of proteasome 20S *α*+*β* and pSTAT3; however, it did not affect the proteasome 20S *α*+*β* mRNA synthesis. Circulating proteasome concentration correlated with tumor tissue proteasome 20S *α*+*β*. STAT3 could occupy the miR-1254 promoter to inhibit transcription, and it could suppressed miR-1254 which targeted PSMD10, promoting proteasome 20S *α*+*β* protein stability. This is a prospective target for developing a new colorectal cancer therapy strategy.

RETRACTED

## 1. Introduction

Colorectal cancer (CRC) is one of the most frequent causes of malignant morbidity and mortality worldwide. More than 1.2 million patients are diagnosed with CRC every year, and more than 600,000 die from the disease [1]. Although vigorous studies have greatly improved the knowledge of colorectal tumorigenesis, the relevant factors that contribute to tumor development and prognosis are still not well determined, which is urgently required for the early detection and treatment of metastatic in CRC.

Increased inflammatory cytokine levels are a distinguishing hallmark of CRC. Interleukin-6 (IL-6) is one of the most prominent protumorigenic cytokines. In the standard IL-6 and STAT3 signaling pathway, IL-6 binding to the cytokine receptor gp130 activates Janus kinase, which results in the phosphorylation of signal transduction, eventually leading to the activation of STAT3; phosphorylation of STAT3 (pSTAT3) gets dimerization and is into the nucleus to regulate target gene transcription [2]. IL-6 has been shown to enhance carcinogenesis and cancer progression, including invasion and metastasis [3].

The ubiquitin-proteasome system (UPS) is the primary mechanism for protein denaturation in eukaryotic cells. UPS contributes to numerous regulatory procedures like cell proliferation, cell cycle, apoptosis, signal transmission, and gene transcription [4–7]. Tumor progression and other diseases are linked to these processes [8–10]. Cancers including basal-like triple-negative breast cancer and multiple myeloma grow faster when the proteasome is activated [11]. On the other hand, proteasome function is essential for antigen production and presentation, which are required for carcinogenesis, immune surveillance, and tumor immunotherapy. Proteasome deregulation may aid tumor cells in evading immune monitoring.

The 26S proteasome consists of 20S core particle and one or two 19S regulatory particles. The UPS in cells is built around the proteasome 20S. The 20S proteasome consists of seven (*β*-subunits) inner rings and seven (*α*-subunits) outer rings arranged in a cylinder shape [12]. Extracellularly, such as in blood serum, the proteasome 20S is found in cells [13]. The oncoprotein gankyrin is encoded by PSMD10, a 26S proteasome non-ATPase regulatory complex [14]. It has been shown that overexpression of this gene occurs in various types of solid tumors. It acts as a tumor promoter, promoting tumor invasiveness and metastasis [15].

MicroRNAs (miRNAs) are a common component of short ncRNA fragments with 22 long and highly conserved nucleotides [16]. Some miRNAs appear to have critical roles in tumor proliferation, apoptosis, differentiation, invasion, and metastasis [17]. miR-1254, a newly discovered miRNA, is dysregulated in several cancers [18]. In colon adenocarcinoma, miR-1254 may operate as a tumor suppressor [19]. However, the interaction between inflammatory cytokines and 20S proteasome in colorectal cancer and its mechanism remains unknown. Therefore, the experiments of vitro and vivo were used in this study to study the role and mechanism of IL-6/STAT3 pathway and 20S proteasome in colorectal cancer.

RETRACTED

## 2. Materials and Methods

### 2.1. Patient Data

The ethical approval for this study was obtained from the “Ethical Committee for Research” of the 3^rd^ Xiangya Hospital, China. All patients gave written or oral consent and were informed about the study's purpose. 90 human CRC tissue samples and nearby normal tissue pairs were provided by Xiangya Hospital, Central South University (Changsha, China). Histopathology verified the finding of colorectal cancer as the cause of the patient's symptoms.  Table 1 summarizes the comprehensive clinicopathological characteristics of the patients who were recruited. A sodium citrate anticoagulant tube was used to collect 4 mL of blood from CRC patients (*n* = 30) and healthy volunteers (*n* = 30). Finally, we selected a cohort of 521 samples taken from primary tumor specimen from the TCGA database in June 2021. Through the TCGA Research Network (http://cancergenome.nih.gov/) established by the NCI and NHGRI, we had obtained the research results.

### 2.2. Immunohistochemistry

Immunohistochemistry (IHC) processes were carried out through the previous method of Dawson et al. [14]. The primary antibody is pSTAT3, proteasome 20S *α*+*β*, and PSMD10 (Abcam, USA). Proteasome 20S *α*+*β* expression and pSTAT3 simultaneously were evaluated by two independent observers. The protein staining was divided into four grades according to staining intensities as follows: 0, 1^+^, 2^+^, and 3^+^. We divided the percentages of protein-positive cells into five categories: 0 (0%), 1 (1–25%), 2 (26–50%), 3 (51–75%), and 4 (76–100%). The immunoreactive score, which is calculated by multiplying the scores of staining intensity and the percentage of positive cells, served as the final score, defined as follows: low proteasome 20S *α*+*β* (staining score < 4) and high proteasome 20S *α*+*β* (staining score ≥ 4), low pSTAT3 (staining score < 6), or high pSTAT3 (staining score ≥ 6) [20, 21].

### 2.3. Detection of Proteasome Plasma Concentration

The ELISA (enzyme-linked immunosorbent assay) assay was used to identify the occurrence of proteasomes in the plasma of CRC patients and healthy participants, according to Sixt and Dahlmann's findings [13]. The microtitration plates were coated with a 1 : 4500 dilution of mice monoclonal antibody to 20S proteasome subunit-6 (HC2) (Biomol International, UK) (pH 7.4). Healthy control plasma was diluted at 1 : 10 and 1 : 5, while all CRC samples at 1 : 1 in PBST-BSA (1% bovine serum albumin, Tween 20, and PBS, 0.1%) were incubated for three hours at RT (room temperature). ELISA standard curve measurements were taken at intervals that fell within the linear part of the curve. Through 20S proteasome protein standards (Biomol International, UK) (concentration range 19.5-2500 ng/mL), standard curves for each microtitration plate were produced (eight linear dilution steps). PBS-T was used to dilute the 20S proteasome (0.1% Tween 20 and PBS). After washing the plates, a rabbit polyclonal antibody to 20S proteasome (Biomol International, UK) (dilution 1 : 4000) was added for 2 hours at room temperature. After four further washing cycles, antigen detection was performed with peroxidase-conjugated mouse anti-rabbit IgG (Sigma-Aldrich, USA) incubated for 1 hour at room temperature. Tetramethylbenzidine (Sigma-Aldrich) was used as a substrate to detect the bound antibodies. Sulphuric acid was used to terminate the process, and odd values at 450 nm were measured. PBS or PBS-T was incubated with BSA (Sigma-Aldrich, Germany) instead of blood plasma to eliminate nonspecific binding wells. In these conditions, no reaction was seen.

RETRACTED

### 2.4. Cell Culture and Transfection

HCT116 and HCT116-R (human colon cancer cell lines) were established in DMEM (1 g/L glucose and 10% fetal calf serum in addition to HEK-293T cells) provided by Invitrogen, USA. The miR-1254 mimic and its negative control (NC) were developed by GenePharma (Shanghai, China). NC for miR-1254 inhibitor and miR-1254 inhibitor was designed and synthesized by GenePharma (Shanghai, China). All sequences of miR-1254 NC, mimic, and inhibitor were as listed in Supplemental Table 1. GenePharma designed and produced vectors containing the PSMD10 3′-UTR sequence or a mutated PSMD10 3′-UTR region (Shanghai, China) (Supplemental Table 2). NC, miR-1254 mimic, and miR-1254 inhibitors were transfected into cells per the manufacturer's guidelines using Lipofectamine 3000 (Invitrogen, Germany).

### 2.5. Cell Treatment

HCT116 and HCT116-R cells were incubated with 20 *μ*M STAT3 inhibitor AG490 (Beyotime, Shanghai, China) at 37°C in 5% CO_2_ for 24 h. HCT116 and HCT116-R cells were also treated with 30 pg/mL IL-6 (Beyotime, Shanghai, China) at 37°C in 5% CO_2_ for 12 h. The cells were treated with the vehicle DMSO as the control.

RETRACTED

### 2.6. Luciferase Reporter Assay

The plasmid of PSMD10 3′-UTR or its mutant sequence (PSMD10 3′-MUT), STAT3 plasmids, the miR-1254 plasmid which knocked out E1 (TTGTTGGAAAA) and E2 (ATTCAAGGAAG) elements (E1-Del/E2-Del) in miR-1254 promoter, and the miR-1254 plasmid which did not knock out E1 and E2 elements (FL) were constructed by Guangzhou Ruibo Biological Co., Ltd. The plasmids of PSMD10 3′-UTR and PSMD10 3′-MUT were cotransfected into HEK-293T cells with the miR-1254 mimic or NC. The plasmids of E1-Del, E2-Del, and FL were cotransfected into HEK-293T cells with the STAT3 plasmids. Following a 48-hour incubation period, luciferase activity was evaluated using the manufacturer's indicated techniques.

### 2.7. RNA Isolation and Quantitative RT-PCR

RNAiso Plus kit was used for total RNA extraction from the cells (TaKaRa, Kyoto, Japan). Reverse transcription was performed using a reverse transcription kit (Fermentas, MD, USA). The One Step SYBR PrimeScript™ TMRT-PCR Kit II was used to amplify the samples using PCR (Takara Bio, Shiga, Japan). miR-1254 expression was standardized to U6 in samples amplified with the ABI ViiATM 7 by Mir-X, miRNA qRT-PCR, and SYBR Kit (Clontech Laboratories, Inc. Japan). As an internal standard for mRNA detection, *α*-actin was used. Supplemental Table 3 contains the qRT-PCR primers.

### 2.8. Western Blot

No cell debris was observed in the cell extracts lysed from treated cells in RIPA buffer after centrifugation. SDS–PAGE was used to separate cell lysates (50 g protein), and PVDF membranes were used to transfer them (Millipore, MA, USA). The following primary antibodies were used to probe the membranes: proteasome 20 *α*+*β*, pSTAT3, *β*-actin, and GADPH (obtained from Abcam, Cambridge, MA, USA).

### 2.9. Immunofluorescence

For 12 hours, HCT116 cells were treated with IL-6 (30 pg/mL) to induce proliferation. Then, the cells were fixed for 10 mins at RT with 4% paraformaldehyde before being labeled with the proteasome 20S *α*+*β* antibody (Abcam, MA, USA).

### 2.10. Chromatin Immunoprecipitation (ChIP) Assay

According to the previously established protocol [22], a Thermo EZ-ChIP Kit was used with phospho-STAT3 and IgG antibodies (Abcam, USA). The associated genomic DNA was observed using a polymerase chain reaction followed by gel electrophoresis (Abcam, USA). Amplification of the pSTAT3-binding areas was achieved using primers specific to the miR-1254 promoter. miR-1254 promoter primers are listed Supplemental Table 4.

### 2.11. Cell Cycle Analysis

The cell cycle was examined through a flow cytometric technique. After transfected cells were fixed in 75% ethanol for 15 minutes, they were stored at -20°C until the next day. The cells were stained with PI staining solution (500 mL, MultiSciences, China), treated with RNAse for 15 minutes at room temperature, and then subjected to a flow cytometric analysis.

RETRACTED

### 2.12. Animal Model Experimentation (Nude Mice)

BALB/c athymic nude mice (male; 4–5 weeks old) received injections under the skin in the right armpit. PBS containing 200 *μ*L of 1 × 10^7^ HCT116 cells was administered subcutaneously. All the mice developed subcutaneous tumors in a week of daily monitoring. Once the tumor had grown to a diameter of about 5 mm, the mice were assigned to one of the three groups randomly using a random number generator: (1) the PBS control group, (2) the IL-6 treatment group, and (3) the miR-1254 mimics with the IL-6 treatment group. Once every four days, 30 mL oligofectamine mixture containing 40 *μ*mol miR-1254 mimics and/or 30 pg/mL IL-6 was used. Tumor volume (*V*, mm [3]) was monitored every 3 days with the caliper and calculated following the formula *V* = (*ab*^2^)/2, wherein *a* is the longest dimension (mm) and *b* is the perpendicular width (mm).

### 2.13. Statistical Analysis

Continuous data were compared using an independent *t*-test. For categorical data analysis, the chi-square test was used. For determinations of survival rates, the Kaplan-Meier survival analysis and log-rank test were performed. The effect of proteasome 20S *α*+*β* and pSTAT3 expression levels and clinic-pathologic characteristics overall survival (OS) were studied using the univariate and multivariate Cox regression. Receiver operating characteristic (ROC) curve was created to assess the circulating proteasome's potential as an early diagnostic biomarker for colorectal cancer. The statistical calculations shown above were carried out using IBM SPSS 26.0 software (IBM, USA). *P* < 0.05 was considered statistically significant.

## 3. Results

### 3.1. The Expression Levels of Proteasome 20S *α*+*β* and pSTAT3 Were Elevated

We used IHC to detect proteasome 20S *α*+*β* and pSTAT3 expression levels in 90 CRC samples and paired neighboring noncancerous tissues. Both markers' expression levels differed significantly between tumor and nearby normal tissues (Figure 1(a)). The expressions of proteasome 20S *α*+*β*, pSTAT3, and STAT3 in the tissues were detected by western blot. The results also showed that the expressions of proteasome 20S *α*+*β* and pSTAT3 in tumor tissues were significantly higher than those in normal tissues, and there was no significant change in the expression of STAT3 (Figure 1(b)). The percentage of cases with high proteasome 20S *α*+*β* staining and high pSTAT3 staining in tumor tissues was 27.78% and 37.78%, respectively. In contrast, the proportion of cases with high proteasome 20S *α*+*β* staining and high pSTAT3 staining in adjacent normal tissues was 4.95% and 14.73%, respectively (*P* < 0.001, Figures 1(c) and 1(d)). Our findings also showed that proteasome 20S *α*+*β* and pSTAT3 expression levels were positively connected with the AJCC (American Joint Committee on Cancer) stages (*P* < 0.01, Figures 1(e) and 1(f)).

RETRACTED

### 3.2. Proteasome 20S *α*+*β* Expression Was Correlated with CRC Progression, as well as pSTAT3

We then looked into the relationship between proteasome 20S *α*+*β* expression and CRC clinicopathological characteristics. It was determined that 90 people with CRC fell into two categories according to proteasome 20S *α*+*β* expression: relative high group (*n* = 25) and relative low group (*n* = 65).  Table 2 summarizes the associations between the expression of the proteasome 20S *α*+*β* and the clinicopathological features of patients with CRC who were studied. The results showed that the amount of proteasome 20S *α*+*β* expression in CRC patients was highly linked with tumor size (*P* < 0.001), lymph node metastasis (*P* = 0.002), distant metastasis (*P* = 0.030), clinical TNM stage (*P* ≤ 0.01), and CEA values (*P* ≤ 0.01). Nonetheless, no significant link was found between proteasome 20S *α*+*β* expression and other clinicopathological parameters such as gender, age, depth of invasion, location, and histological grade (*P* > 0.05). Our findings suggested that increased proteasome 20S *α*+*β* expression may be linked to CRC progression.

Furthermore, we classified all cases based on the pSTAT3 expression pattern into low pSTAT3 (57 cases) or high pSTAT3 categories (33 cases). We discovered that proteasome 20S *α*+*β* expression was significantly higher in patients with high pSTAT3 staining than in cases with low pSTAT3 staining (*P* ≤ 0.01, Table 2). As a result, the proportion of patients with high proteasome 20S *α*+*β* staining increased from 10.53% in the low pSTAT3 group to 57.58% in the high pSTAT3 group. The percentage of instances with poor proteasome 20S *α*+*β* expression, on the other hand, reduced from 89.47% in the low pSTAT3 group to 42.42% in the high pSTAT3 group.

### 3.3. Upregulated Expression Levels of Proteasome 20S *α*+*β* and pSTAT3 Associated with Poor Prognosis in CRC Patients

The Kaplan-Meier and log-rank tests were used to analyze the indicator expression-prognosis connection. The findings demonstrated that the OS in CRC patients with overexpression of proteasome 20S *α*+*β* and pSTAT3 was poorer than in those with lower expression of the two proteins (*P* < 0.001 and *P* = 0.0022, respectively) (Figures 2(a) and 2(b)). We also looked at the relationship between proteasome 20S *α*+*β* and pSTAT3 with overall survival. The group with higher levels of proteasome 20S *α*+*β* and pSTAT3 expression simultaneously had a considerably worse prognosis than the group with lower levels of both proteins (*P* < 0.001) (Figure 2(c)).

RETRACTED

Univariate analysis showed six predictive variables for poor survival: tumor size (*P* < 0.001), lymph node metastasis (*P* < 0.001), histological grade (*P* = 0.004), TNM stage (*P* ≤ 0.01), pSTAT3 expression (*P* = 0.003), and proteasome 20S *α*+*β* expression (*P* ≤ 0.01) (Table 3). Multivariate analysis revealed that proteasome 20S *α*+*β* expression (*P* ≤ 0.01), as well as TNM stage (*P* = 0.029), was an independent predictor of poor prognosis in CRC patients (Table 3). In conclusion, our data suggested that elevated expression of proteasome 20S *α*+*β* might serve a role in the formation, development, and prognosis of CRC patients with IL-6/STAT3 activation.

### 3.4. Circulating Proteasome Was Positively Correlated with Tumor Tissue Proteasome 20S *α*+*β* and Had Potential Diagnostic Value in CRC Patients

The circulating proteasome concentrations were considerably more significant in patients with colorectal cancer than in healthy controls (*P* < 0.001) (Figure 3(a)). As illustrated in Figure 3(b), circulating proteasome associated favorably with tumor tissue proteasome 20S *α*+*β* in 30 patient samples (*r* = 0.0.6582, *P* < 0.001).

To further investigate the circulating proteasome's potential diagnostic usefulness, ROC curve was created to assess the circulating proteasome's potential as an early diagnostic biomarker for colorectal cancer. As illustrated in Figure 3(c), ROC analysis revealed that the optimal cut-off level for circulating proteasome to diagnose CRC was 462 ng/mL (area under the curve (AUC): 0.949, 95% CI: 0.859–0.923, *P* < 0.001), indicating that circulating proteasome may be a promising tumor marker for CRC diagnosis.

### 3.5. IL-6/STAT3 Induced Upregulated Expression of Proteasome 20S *α*+*β*

To investigate the probable mechanism underlying the increased proteasome 20S *α*+*β* expression in response to IL-6/STAT3 activation, we employed IL-6 as an inflammatory stimulant. Proteasome 20S *α*+*β* protein levels were elevated in HCT116 cell lines following IL-6 stimulation (Figures 4(a) and 4(b)). However, IL-6 stimulus did not significantly affect proteasome 20S *α*+*β* mRNA level (Figures 4(c) and 4(d)), indicating that IL-6 stimulus did not affect proteasome 20S *α*+*β* mRNA synthesis.

### 3.6. miR-1254 Targeting PSMD10 Promoted Protein Degradation of Proteasome 20S *α*+*β*

The NPInter database (http://bigdata.ibp.ac.cn/npinter4/interaction/ncRI-40969679/) provides insight into the miR-1254-PSMD10 interaction molecules. The miR-1254 levels remained considerably lower in colorectal cancer lesion tissues than in neighboring nontumor tissues (Figure 5(a)). Simultaneously, we demonstrate that PSMD10 expression is considerably more in CRC lesions than in surrounding tissues (Figure 5(b)). According to the TCGA database, PSMD10 expression is negatively correlated with miR-1254 (Figure 5(c)). To investigate the role of miR-1254 in HCT116 cells, we transfected with various amounts of miR-1254 mimics and its inhibitor to the colon cancer cell line HCT116. Finally, 40 *μ*M miR-1254 mimics and 40 *μ*M miR-1254 inhibitors were chosen as the transfection conditions for future transfection (Figures 5(d) and 5(e)). To determine whether miR-1254 directly attenuates the expression of PSMD10 by interaction with its 3′-UTR, PSMD10 3′-UTR luciferase vectors encoding the miR-1254 reactive fragment or a mutated sequence were used to conduct luciferase assays in HEK-293 cells. Cotransfection of the plasmids with miR-1254 mimics or NC showed a 50.7% decrease of luciferase activity in cells simultaneously transfected with PSMD10 3′-UTR reporter plasmids and miR-1254 mimic. In contrast, in cells transfected with plasmids containing a mutated version of the miR-1254 binding site of PSMD10 3′-UTR, the miR-1254 mimics were unsuccessful in decreasing luciferase activity (Figure 5(f)). In CRC cell HCT116, miR-1254 inhibitors or mimics, as well as their NC, were transfected. PSMD10 expression was downregulated in response to miR-1254 mimic. In comparison, CRC cells were transfected with miR-1254 inhibitors. PSMD10 expression was increased. The western blot examination also demonstrated that miR-1254 mimic reduced proteasome 20S *α*+*β*. Transfection of miR-1254 inhibitor increased proteasome 20S *α*+*β* expression (Figure 5(g)). Following that, 40 *μ*M miR-1254 mimics were chosen as the transfection conditions. Proteasome 20S *α*+*β* protein levels in colon cancer HCT116 cell lines were found to be reduced in a time-dependent way following miR-1254 mimic stimulation (Figure 5(h)).

RETRACTED

### 3.7. STAT3 Could Activate miR-1254 Transcription

We uncovered two potential STAT3-binding sites near the miR-1254 promoter region through bioinformatics analysis (Figure 6(a)). After treating HCT116 cells with the STAT3 inhibitor AG490 for 12 h, it was observed that the expression of pSTAT3 was significantly lower than that in the NC group, indicating that the inhibition of STAT3 was successful (Figure 6(b)). Then, we looked at whether STAT3 could influence miR-1254 expression. A qRT-PCR experiment revealed that IL-6 significantly reduced miR-1254 transcription, whereas IL-6+AG490 significantly raised miR-1254 levels (Figure 6(c)). Luciferase assay indicated the miR-1254 promoter was significantly repressed by STAT3 and was transactivated by STAT3 inhibitor AG490 treatment (Figures 6(d) and 6(e)). The two predicted STAT3-binding sites were removed independently to determine which element was required for STAT3-mediated miR-1254 production. The STAT3 was almost unsuccessful in regulating miR-1254 transcriptional activity in the absence of the E1 element indicating that the E1 element was required for STAT3 to regulate miR-1254 transcription (Figure 6(f)). For confirmation of these findings, a chromatin immunoprecipitation (ChIP) test was performed using a pSTAT3 antibody, followed by PCR detection. STAT3 could bind with the miR-1254 promoter and was abundant in the E1 region (-1160~-1150 bp), as seen in Figure 6(g).

### 3.8. Differential Effects on Cell Cycle of miR-1254

Flow cytometry was used to determine cell cycle distribution (Figures 7(a)–7(d)). The results showed that HCT116 cells treated with miR-1254 mimicked a longer cell cycle in the G0/G1 phase (Figure 7(e)), but HCT116-R cells transfected with the miR-1254 inhibitor exhibited the reverse trend (Figure 7(f)).

### 3.9. In Vivo miR-1254 Targeting PSMD10 Mediated Proteasome 20S *α*+*β* Stability

We employed a xenograft mouse model to investigate miR-1254's role in cancer growth. IL-6 therapy enhanced xenograft tumor growth, whereas miR-1254 combined with IL-6 treatment significantly suppressed xenograft tumor growth (Figures 8(a)–8(c)). The levels of miR-1254 expression in implanted tumors were investigated (Figure 8(d)). The tumor tissues were excised and stained with immunohistochemistry, showing a substantial increase in p-STAT3, PSMD10, and proteasome 20S *α*+*β* in the IL-6 group over the PBS group. In contrast, this result was reversed when miR-1254 mimics were paired with IL-6 administration (Figure 8(e)).

## 4. Discussion

The present investigation confirmed that IL-6/STAT3 activation boosted proteasome 20S *α*+*β* expression in CRC. The progression of CRC was linked to increased expression of the proteasome 20S *α*+*β*. Patients with higher levels of proteasome 20S *α*+*β* expression and activation of IL-6/STAT3 had a shorter OS than those with lower levels of proteasome 20S *α*+*β* expression and inactivation of IL-6/STAT3. In the multivariate Cox regression studies, the proteasome 20S *α*+*β* expression and the TNM stage were independent predictive risk factors for CRC patients. Furthermore, we found that IL-6 stimulation significantly increased the expression of the proteasome 20S *α*+*β* in vitro. We looked into the 20S proteasomes found in the blood serum of CRC patients. There was also a rise in circulating proteasome concentrations in blood serum, which positively correlated with tumor tissue expression levels of proteasome 20S *α*+*β*. We discovered that IL-6 stimulation had no effect on the synthesis of 20S mRNA for the proteasome. To our surprise, we discovered that STAT3 signaling pathway suppressed miR-1254 transcription, which in turn increased the production of PSMD10, a protein essential for proteasome 20S stability. We also discovered that STAT3 might bind to the miR-1254 promoter, which would make it harder for the gene to be transcribed.

RETRACTED

The UPS (ubiquitin-proteasome system) is involved in the breakdown of intracellular proteins. The 20S proteasome is essential for intracellular UPS, and the proteasome 20S plays a significant role in carcinogenesis and tumor progression [23]. Proteasome 20S *α*+*β* expression levels were elevated in CRC patients. They were highly linked with CEA values, clinical TNM stage, far-off metastasis, lymph node metastasis, and tumor size, indicating that this protein played a critical role in CRC progression. In addition, we discovered that elevated levels of proteasome 20S *α*+*β* expression were closely linked to pSTAT3 in CRC patients. When STAT3 has been phosphorylated (tyrosine 705), it may go to the nucleus, regulating gene transcription via the IL-6/STAT3 pathway [24]. pSTAT3, which is overexpressed in a variety of cancers, is considered an oncogene [25, 26]. Additionally, it may play a substantial role in the course of malignancy [27].

Our investigation perceived a considerable increase in pSTAT3 expression in tumor tissues compared to surrounding normal tissues. Additionally, IL-6 enhances the expression of the proteasome 20S *α*+*β in vitro*, implying that pSTAT3 possibly will play a crucial part in promoting proteasome20S *α*+*β* expression.

Proteasome 20S *α*+*β* and pSTAT3 were found to be predictive of poor prognosis in patients with colorectal cancer. The Kaplan-Meier analysis demonstrated that individuals with CRC who overexpressed proteasome 20S *α*+*β* and pSTAT3 had a shorter OS than those who have lower expression of the two proteins. The Cox proportional hazard modeling was used. The results established that elevated proteasome 20S *α*+*β* expression was an independent marker of poor overall survival of CRC patients.

Surprisingly, human blood contains circulating proteasome 20S [28]. An increasing body of evidence indicates that cancer patients have greater plasma proteasome concentrations than healthy controls [29–31]. In this investigation, we observed an increase in the expression of circulating proteasome 20S *α* + *β* in individuals with colorectal cancer. A substantial association among the levels of the proteasome in plasma and tumor tissues was observed. The ROC curves demonstrated a significant difference between the plasma and control groups. As a result, the circulating proteasome had the highest diagnostic power for CRC detection, implying that circulating proteasome 20S *α*+*β* may be a useful tumor marker for CRC diagnosis.

RETRACTED

The current work discovered that PSMD10 expression is inversely linked with miR-1254 expression in the TCGA database. A dual-luciferase reporter test demonstrated that miR-1254 was capable of binding selectively to the 3′-UTR of PSMD10. PSMD10, called proteasome non-ATPase regulatory subunit 10 or gankyrin, containing a seven ankyrin repeat [32]. PSMD10 was viewed as a subunit of 19S complex to regulate the 26S proteasome [33]. It is upregulated in a variety of human cancers. It acted as a tumor promoter, promoting tumor invasiveness and metastasis [34]. The overexpression of miR-1254 resulted in a cell cycle arrest in the G1-phase and reduced cells in the S-phase. This finding suggests that miR-1254 may function as a tumor suppressor in colon cancer. Proteasome 20S *α*+*β* expression was upregulated in reaction to an increase in PSMD10. We employed miR-1254 mimics to transfect HCT116 cell lines and discovered that miR-1254 mimics dramatically lowered the stability of proteasome 20S *α*+*β* protein levels as compared to the control group, which indicates that PSMD10 aided in the stabilization of the proteasome 20S *α*+*β* by reducing miR-1254.

We found a novel miR-1254 promoter-binding protein, STAT3, in this investigation. By directly occupying the miR-1254 promoter region inside the 1160~-1150 bp motif, active STAT3 decreases miR-1254 production. Previous research established that overexpression of PSMD10 improves signal transducer and initiation of transcription STAT3-phosphorylation and facilitates pSTAT3 nuclear translocation. STAT3 plays a critical role in cancer growth. It regulates many genes involved in cell proliferation, immunosuppression, angiogenesis, and invasion [35]. Meanwhile, we discovered that active STAT3 inhibited miR-1254 expression to increase PSMD10 production. We demonstrated that overexpression of miR-1254 cases resulted in expression levels downregulated in the PSMD10 and proteasome 20S *α*+*β*, which inhibited tumor development in model mouse xenograft compared to IL-6 activation.

In conclusion, we discovered in this study that increasing proteasome 20S *α*+*β* expression levels had a strong correlation with pSTAT3 in patients with colorectal cancer. Additionally, these increased proteasome 20S *α*+*β* expressions were related to CRC development and clinical outcome. Additionally, we observed a substantial upregulation of proteasome 20S *α*+*β* expression in vitro in response to IL-6 stimulation. We studied the 20S proteasomes found in the blood serum of patients with colorectal cancer. Proteasome concentrations in blood serum also rose and were associated positively with proteasome 20S *α*+*β* expression levels in tumor tissues. Nevertheless, IL-6 did not affect the proteasome involved in the synthesis of 20S *α*+*β* mRNA. We established a link between miR-1254 and PSMD10 and demonstrated that miR-1254 via targeting PSMD10 regulated the cell cycle. Increased PSMD10 expression enhanced proteasome 20S *α*+*β* protein stability. Additionally, we demonstrated that STAT3 could bind to the miR-1254 promoter, inhibiting its transcription. Finally, our research showed that miR-1254 targeting PSMD10 impacted protein stability of proteasome 20S *α*+*β*, a prospective target for developing a new colorectal cancer therapy strategy.

RETRACTED

## Figures and Tables

**Figure 1:** The expressions of proteasome 20S *α*+*β* and pSTAT3 were elevated in CRC patients. (a) Representative pictures of the proteasome 20S *α*+*β* and pSTAT3 in tumor and normal tissues. (b) The expression of proteasome 20S *α*+*β*, pSTAT3, and STAT3 in tumor and normal tissues. The scale bar measures 50 *μ*m. (c and d) Differences in pSTAT3 (c) and proteasome expression 20S *α*+*β* (d) were found in the tumor and surrounding normal tissues (*P* < 0.001 and *P* < 0.001, respectively, *χ*^2^ test). (e and f) The expressions of proteasome 20S *α*+*β* (e) and pSTAT3 (f) were similarly positively linked with AJCC stages (*P* < 0.01 and *P* < 0.01, respectively, *χ*^2^ test).

**Figure 2:** Patients with colorectal cancer (CRC) were assessed through the Kaplan-Meier survival curves according to proteasome 20S *α*+*β* (a), pSTAT3 (b), and combined proteasome 20S *α*+*β* and pSTAT3 status (c). The *P* value was determined using the log-rank test (*P* < 0.05).

**Figure 3:** (a) ELISA analysis was performed on a total of 30 plasma trials from CRC patients and 30 healthy controls. The data were reported as mean ± SD and evaluated using the Student's *t*-test. ^∗∗∗^*P* < 0.001 is indicated. (b) Plasma and tumor tissue proteasome levels were compared in patients with colorectal cancer. *r* = 0.6582 indicates a substantial association between the levels of proteasome expression in plasma and tumor tissue. (c) ROC curve discriminates using a circulating proteasome level between CRC patients and the control group. The graphs depicted the area under the curve (AUC).

RETRACTED

**Figure 4:** IL-6/STAT3 increased the expression of the proteasome 20S *α*+*β*. IL-6 (30 pg/mL) or PBS was used to activate HCT116 cells, taking samples at the indicated time. (a) Cells were fixed and stained as described: proteasome 20S *α*+*β* (green) and DAPI (blue). (b) Proteasome 20S *α*+*β* and GADPH immunoblots were generated from lysates. (c and d) For 12 hours, HCT116 cells were stimulated with either IL-6 (30 pg/mL). qRT-PCR was used to determine the proteasome 20S *α* (PSMA1-A7) and proteasome 20S *β* (PSMB1-B7) mRNA levels.

**Figure 5:** miR-1254 targeting PSMD10 promoted protein degradation of proteasome 20S *α*+*β*. (a) RT-PCR analysis demonstrates that miR-1254 levels decrease in colorectal cancer lesions relative to the surrounding tissues. (b) The analysis of RT-PCR demonstrates that PSMD10 levels are elevated in CRC lesions relative to surrounding tissues in paired tissue samples. (c) In the tissue sample of TGGA databases, a negative connection between PSMD10 and miR-1254 transcription was found. (d) HCT116 cells were transfected with negative control (NC) and miR-1254 mimics at varying doses (20 *μ*M and 40 *μ*M). qRT-PCR was used to detect miR-1254 expression. (e) Lip2000 was used to transfect HCT116 with negative control (NC) and different concentrations (20 *μ*M and 40 *μ*M) of miR-1254 inhibitor. qRT-PCR was used to detect miR-1254 expression. (f) miR-1254 inhibited the luciferase activity of the PSMD10 3′-UTR reporter plasmid by 50.7% in HEK-293 cells. (g) Western blot investigation has shown that PSMD10 expression was modulated following transfection with miR-1254 mimics and inhibitors in HCT116 cells. (h) HCT116 cells were transfected with miR-1254 mimics for 12 h; at that time, they were administered with different doses of cycloheximide (CHX) and harvested at the given time points. PSMD10 and proteasome 20S *α*+*β* were immunoblotted from lysates. ^∗∗∗^*P* < 0.001, ^∗∗^*P* < 0.01, and ^∗^*P* < 0.05.

**Figure 6:** STAT3 could inactivate the transcription of miR-1254 (a). The classic STAT3-binding motif (JASPAR Database) and two putative STAT3 responsive elements (E1 and E2) in the miR-1254 promoter region are depicted in a schematic diagram. TSS refers to miR-1254's transcriptional start point. (b) HCT116 cells were treated with STAT3 inhibitor AG490 at a concentration of 20 *μ*M. The expressions of pSTAT3 were analyzed by western blot. (c) HCT116 cells were treated with IL-6 or AG490. miR-1254 mRNA levels were analyzed by RT-PCR. (d) When the cells were transfected with STAT3 plasmids, the luciferase assay was employed to determine miR-1254 promoter transcriptional activity. (e) miR-1254 promoter activity when cells were treated with AG490. (f) Two putative STAT3-binding sites in the miR-1254 promoter were removed, labeled E1-Del and E2-Del. When STAT3 expression was driven in HCT116 cells, the transcriptional activity of the two miR-1254 promoter deletion mutants was assessed through luciferase assay. (g) ChIP experiments revealed that STAT3 is linked to the miR-1254 promoter's E1 element. As a negative control, IgG was used. ^∗∗∗^*P* < 0.001, ^∗∗^*P* < 0.01, and ^∗^*P* < 0.05.

RETRACTED

**Figure 7:** Effects of the miR-1254 variation on cell cycle distribution. (a–d) For 48 hours, the cells were transfected with the indicated miR-1254 mimics (HCT116) or inhibitors (HCT116-R). After that, the cells were extracted, and a cell cycle was measured using a flow cytometry test. The flow cytometry experiment of treated cells is shown above, with a representative picture. (e) HCT116 cells transfected with miR-1254 mimics simulate an extended G0/G1 cell cycle. (f) HCT116-R cells treated with a miR-1254 inhibitor shorted cell cycle progression in the G0/G1 phase. ^∗∗∗^*P* < 0.001, ^∗∗^*P* < 0.01, and ^∗^*P* < 0.05.

**Figure 8:** miR-1254 targeting PSMD10 mediated proteasome 20S *α*+*β* degradation *in vivo*. The nude mice had injected with the HCT116 cells subcutaneously. When the tumor size reached around 5 mm, the mice were separated into three groups randomly. PBS, IL-6, and IL-6+miR-1254s were injected intratumorally into mice. The animals were slaughtered four weeks following the treatment, and their tumor growth was monitored. (a) Comparison of excised tumor size in each group. (b) The weight of tumor for the 4 xenograft tumor groups. (c) The curves of tumor growth volume of the three xenograft tumor groups. (d) RT-PCR was used to investigate the expression levels of miR-1254 in the implanted tumors. (e) Immunohistochemistry was used to detect the expression of p-STAT3, PAMD10, and proteasome 20S *α*+*β* in xenograft tumors groups. The scale bar measures 50 *μ*m. All data were presented as means ± SD, with ^∗∗^*P* < 0.01 compared to the PBS group and ^∗∗∗^*P* < 0.01 compared to the PBS group.

**Table 1:** Clinicopathologic characteristics in 90 CRC patients.

Variables	Cases (%)
Gender	
Male	42 (46.7)
Female	48 (53.3)
Age (years)	
≤60	29 (32.2)
>60	61 (67.8)
Size	
≤5 cm	43 (47.8)
>5 cm	47 (52.2)
Depth of invasion	
≤pT2	13 (14.4)
≥pT3	77 (85.6)
Lymph node metastasis	
No	59 (65.6)
Yes	31 (34.4)
Distant metastasis	
No metastasis	85 (94.4)
Metastasis	5 (5.6)
Localization	
Proximal colon	14 (15.6)
Distal colon	76 (84.4)
Histological grade	
Well	6 (6.7)
Moderately	70 (77.8)
Poorly	14 (15.6)
TNM stage	
I and II	57 (63.3)
III and IV	33 (36.7)
CEA (*μ*g/L)	
≥5	54 (60.0)
<5	36 (40.0)

RETRACTED

**Table 2:** Correlation between proteasome 20S *α*+*β* expression and clinicopathologic characteristics in 90 CRC patients.

Variables	Proteasome 20S *α*+*β* expression			
	Total	Low	High	*P* value
Gender				0.432
Male	42	32 (76.2%)	10 (23.8%)	
Female	48	33 (68.8%)	15 (31.2%)	
Age (years)				0.595
≤60	29	22 (75.9%)	7 (24.1%)	
>60	61	43 (70.5%)	18 (29.5%)	
Size				0.001^∗∗∗^
≤5 cm	43	38 (88.4%)	5 (11.6%)	
>5 cm	47	27 (57.4%)	20 (42.6%)	
Depth of invasion				0.457
≤pT2	13	11 (84.6%)	2 (15.4%)	
≥pT3	77	54 (70.1%)	23 (29.9%)	
Lymph node metastasis				0.002^∗∗^
No	59	49 (83.1%)	10 (16.9%)	
Yes	31	16 (51.6%)	15 (48.4%)	
Distant metastasis				0.030^∗^
No metastasis	85	64 (75.3%)	21 (24.7%)	
Metastasis	5	1 (20.0%)	4 (80.0%)	
Localization				0.367
Proximal colon	14	12 (85.7%)	2 (14.3%)	
Distal colon	76	53 (69.7%)	23 (30.3%)	
TNM stage				≤0.01
I and II	57	49 (86.0%)	8 (14.0%)	
III and IV	33	16 (48.5%)	17 (51.5%)	
Histological grade				0.140
Well	6	5 (83.3%)	1 (16.7%)	
Moderately	70	53 (75.7%)	17 (24.3%)	
Poorly	14	7 (50.0%)	7 (50.0%)	
CEA (*μ*g/L)				≤0.01
≥5	54	47 (87.0%)	7 (13.0%)	
<5	36	18 (72.2%)	18 (27.8%)	
pSTAT3				≤0.01
Low	57	51 (89.47%)	6 (10.53%)	
High	33	14 (42.42%)	19 (57.58%)	

^∗^ *P* < 0.05, ^∗∗^*P* < 0.01, and ^∗∗∗^*P* < 0.001.

**Table 3:** Univariate and multivariate Cox regression analyses of overall survival in 90 CRC patients.

Variables	Univariate analysis (Cox: enter)			Multivariate analysis (Cox: forward conditional)		
	HR	95% CI	p	HR	95% CI	*P*
Gender						
Male versus female	0.770	0.389–1.526	0.454			
Age (years)						
≤60 versus >60	1.200	0.574–2.511	0.628			
Size (cm)						
≤5 versus >5	3.471	1.616–7.456	0.001			
Depth of invasion						
≤pT2 versus ≥pT3	1.945	0.594–6.365	0.271			
Lymph node metastasis						
No versus yes	3.197	1.619–6.310	0.001			
Distant metastasis						
No metastasis versus metastasis	2.841	0.996–8.105	0.051			
Localization						
Proximal versus distal	1.131	0.438–2.922	0.799			
Histological grade						
Well and moderate versus poor	2.824	1.385–5.760	0.004			
TNM stage						
I and II versus III and IV	3.866	1.927–7.758	≤0.01	2.423	1.093–5.376	0.029
CEA						
≥5 versus <5	1.081	0.546–2.141	0.823			
pSTAT3						
Low versus high	2.762	1.397–5.458	0.003			
Proteasome 20S *α*+*β*						
Low versus high	5.335	2.679–10.624	≤0.01	4.214	2.058–8.628	≤0.01

HR: hazard ratio; 95% CI: 95% confidence interval.

## Data Availability

The data used to support the findings of this study are available from the corresponding author upon request.

## Supplementary Materials

Supplementary 1 Supplemental Table 1: sequences of miR-1254 NC, mimic, and inhibitor.

RETRACTED

Supplementary 2 Supplemental Table 2: primer sequences used for ChIP assay.

Supplementary 3 Supplemental Table 3: primer list for real-time PCR.

Supplementary 4 Supplemental Table 4: primer sequences used for ChIP assay.

## References

[1] Dekker E., Tanis P. J., Vleugels J., Kasi P. M., Wallace M. B. (2019). Colorectal cancer. *Lancet*.

[2] Sansone P., Bromberg J. (2012). Targeting the interleukin-6/Jak/stat pathway in human malignancies. *Journal of Clinical Oncology*.

[3] Taniguchi K., Karin M. (2014). IL-6 and related cytokines as the critical lynchpins between inflammation and cancer. *Seminars in Immunology*.

[4] Guillaume B., Chapiro J., Stroobant V. (2010). Two abundant proteasome subtypes that uniquely process some antigens presented by HLA class I molecules. *Proceedings of the National Academy of Sciences of the United States of America*.

[5] Voges D., Zwickl P., Baumeister W. (1999). The 26S proteasome: a molecular machine designed for controlled proteolysis. *Annual Review of Biochemistry*.

[6] Glickman M. H., Ciechanover A. (2002). The ubiquitin-proteasome proteolytic pathway: destruction for the sake of construction. *Physiological Reviews*.

[7] Adams J. (2003). The proteasome: structure, function, and role in the cell. *Cancer Treatment Reviews*.

[8] Heubner M., Wimberger P., Dahlmann B. (2011). The prognostic impact of circulating proteasome concentrations in patients with epithelial ovarian cancer. *Gynecologic Oncology*.

[9] Spirina L. V., Yunusova N. V., Kondakova I. V. (2012). Association of growth factors, HIF-1 and NF-*κ*B expression with proteasomes in endometrial cancer. *Molecular Biology Reports*.

[10] Jalovecka M., Hartmann D., Miyamoto Y. (2018). Validation of Babesia proteasome as a drug target. *International Journal for Parasitology: Drugs and Drug Resistance*.

[11] Marcotte R., Sayad A., Brown K. R. (2016). Functional genomic landscape of human breast cancer drivers, vulnerabilities, and resistance. *Cell*.

[12] Kopp F., Hendil K. B., Dahlmann B., Kristensen P., Sobek A., Uerkvitz W. (1997). Subunit arrangement in the human 20S proteasome. *Proceedings of the National Academy of Sciences of the United States of America*.

[13] Sixt S. U., Dahlmann B. (2008). Extracellular, circulating proteasomes and ubiquitin - incidence and relevance. *Biochimica et Biophysica Acta*.

[14] Dawson S., Apcher S., Mee M. (2002). Gankyrin is an ankyrin-repeat oncoprotein that interacts with CDK4 kinase and the S6 ATPase of the 26 S proteasome. *The Journal of Biological Chemistry*.

[15] Liu Y., Zhang J., Qian W. (2014). Gankyrin is frequently overexpressed in cervical high grade disease and is associated with cervical carcinogenesis and metastasis. *PLoS One*.

RETRACTED

[16] Bartel D. P. (2004). MicroRNAs: genomics, biogenesis, mechanism, and function. *Cell*.

[17] Ameres S. L., Zamore P. D. (2013). Diversifying microRNA sequence and function. *Nature Reviews. Molecular Cell Biology*.

[18] Lu M., Chen W. H., Wang C. Y., Mao C. Q., Wang J. (2017). Reciprocal regulation of miR-1254 and c-Myc in oral squamous cell carcinoma suppresses EMT-mediated metastasis and tumor-initiating properties through MAPK signaling. *Biochemical and Biophysical Research Communications*.

[19] Chu Y. M., Peng H. X., Xu Y. (2017). MicroRNA-1254 inhibits the migration of colon adenocarcinoma cells by targeting PSMD10. *Journal of Digestive Diseases*.

[20] Castillo S. D., Angulo B., Suarez-Gauthier A. (2010). Gene amplification of the transcription factor DP1 and CTNND1 in human lung cancer. *The Journal of Pathology*.

[21] Ren W., Shen S., Sun Z. (2016). Jak-STAT3 pathway triggers DICER1 for proteasomal degradation by ubiquitin ligase complex of CUL4A^DCAF1^ to promote colon cancer development. *Cancer Letters*.

[22] Ross J., Bottardi S., Bourgoin V. (2009). Differential requirement of a distal regulatory region for pre-initiation complex formation at globin gene promoters. *Nucleic Acids Research*.

[23] Golab J., Bauer T. M., Daniel V., Naujokat C. (2004). Role of the ubiquitin-proteasome pathway in the diagnosis of human diseases. *Clinica Chimica Acta*.

[24] Sriuranpong V., Park J. I., Amornphimoltham P., Patel V., Nelkin B. D., Gutkind J. S. (2003). Epidermal growth factor receptor-independent constitutive activation of STAT3 in head and neck squamous cell carcinoma is mediated by the autocrine/paracrine stimulation of the interleukin 6/gp130 cytokine system. *Cancer Research*.

[25] Lee M., Hirpara J. L., Eu J. Q. (2019). Targeting STAT3 and oxidative phosphorylation in oncogene-addicted tumors. *Redox Biology*.

[26] Attili I., Karachaliou N., Bonanno L. (2018). STAT3 as a potential immunotherapy biomarker in oncogene-addicted non-small cell lung cancer. *Therapeutic Advances in Medical Oncology*.

[27] Alvarez J. V., Febbo P. G., Ramaswamy S., Loda M., Richardson A., Frank D. A. (2005). Identification of a genetic signature of activated signal transducer and activator of transcription 3 in human tumors. *Cancer Research*.

[28] Wada M., Kosaka M., Saito S., Sano T., Tanaka K., Ichihara A. (1993). Serum concentration and localization in tumor cells of proteasomes in patients with hematologic malignancy and their pathophysiologic significance. *The Journal of Laboratory and Clinical Medicine*.

[29] Stoebner P. E., Lavabre-Bertrand T., Henry L. (2005). High plasma proteasome levels are detected in patients with metastatic malignant melanoma. *The British Journal of Dermatology*.

RETRACTED

[30] Lavabre‐Bertrand T., Henry L., Carillo S. (2001). Plasma proteasome level is a potential marker in patients with solid tumors and hemopoietic malignancies. *Cancer*.

[31] Dutaud D., Aubry L., Henry L. (2002). Development and evaluation of a sandwich ELISA for quantification of the 20S proteasome in human plasma. *Journal of Immunological Methods*.

[32] Higashitsuji H., Itoh K., Nagao T. (2000). Reduced stability of retinoblastoma protein by gankyrin, an oncogenic ankyrin-repeat protein overexpressed in hepatomas. *Nature Medicine*.

[33] Fu X. Y., Wang H. Y., Tan L., Liu S. Q., Cao H. F., Wu M. C. (2002). Overexpression of p28/gankyrin in human hepatocellular carcinoma and its clinical significance. *World Journal of Gastroenterology*.

[34] Fu J., Chen Y., Cao J. (2011). p28GANK overexpression accelerates hepatocellular carcinoma invasiveness and metastasis via phosphoinositol 3-kinase/AKT/hypoxia-inducible factor-1*α* pathways. *Hepatology*.

[35] Yu H., Lee H., Herrmann A., Herrmann A., Buettner R., Jove R. (2014). Revisiting STAT3 signalling in cancer: new and unexpected biological functions. *Nature Reviews. Cancer*.

